This article has been retracted.

# Proteomics Analysis of Serum Proteins in Gestational Diabetes

**DOI:** 10.1155/2021/4724590

**Published:** 2021-11-02

**Authors:** Jianhua Li, Lin Lu, Xinping Xie, Xiaofeng Dai, Shan Zheng, Lihong Chen

**Affiliations:** Department of Obstetrics and Gynecology, The First Affiliated Hospital of Fujian Medical University, Fuzhou, Fujian 350005, China

## Abstract

**Objective:**

The purpose of this study was to screen serum proteins for biomarkers of gestational diabetes mellitus (GDM) and to investigate its pathogenesis by analyzing the differences in serum proteomics between pregnant women with GDM and healthy pregnant women.

**Methods:**

Patients who were admitted to the First Affiliated Hospital of Fujian Medical University from June 2019 to January 2020 were included. According to the medical history and the results of the 75 g oral glucose tolerance test (OGTT), they were divided into the normal pregnant women group and GDM pregnant women group. The serum of two groups of patients was collected. High performance liquid chromatography-mass spectrometry was used to identify differentially expressed serum proteins between pregnant women with GDM and healthy pregnant women, and bioinformatics analysis was then performed on the identified proteins.

**Results:**

A total of 1152 quantifiable proteins were detected; among them, 15 were upregulated in serum of GDM pregnant women, while 26 were downregulated. The subsequent parallel reaction monitoring (PRM) assay validated the expression levels of 12 out of 41 differentially expressed proteins. Moreover, bioinformatics analysis revealed that the differentially expressed proteins are involved in multiple biological processes and signaling pathways related to the lipid metabolism, glycan degradation, immune response, and platelet aggregation.

**Conclusions:**

This study identified 41 serum proteins with differential expression between pregnant women with GDM and healthy pregnant women, providing new candidate molecules for elucidating GDM pathogenesis and screening therapeutic targets.

## 1. Introduction

Gestational diabetes mellitus (GDM) is defined as a varying degree of glucose tolerance disorder that occurs or is first recognized during pregnancy [1]. As the most common complication of pregnancy, GDM seriously threatens the short-term and long-term health of mothers and their offspring, becoming a growing public health problem worldwide [2]. Although GDM has been shown to be related to adipokines [3], inflammation [4], insulin resistance, and cellular dysfunction [5], its pathogenesis has not yet to be fully elucidated. At present, the clinical diagnosis of GDM is conducted mainly based on the analysis of hyperglycemia and the study of adverse pregnancy outcomes using criteria issued by the International Association of Diabetes and Pregnancy Study Groups. However, this diagnosis method has certain defects, causing a misdiagnosis of mild glucose intolerance as GDM [6]. Thus, pathogenesis studies and identification of new diagnostic markers could make GDM diagnosis more accurate and help to control the occurrence and development of this disease.

Proteomics, which has been widely used in basic research and clinical diagnosis of human diseases, involves analysis, characterization, and classification of all protein in a genome [7]. In particular, differential proteomics provides a powerful technique for identifying different molecules based on comparison of the changes in protein levels between samples, investigating disease-related differential proteomics as a whole, and searching for protein markers of diseases. With the help of differential proteomics, the pathogenesis of GDM can be further explored due to the fact that the protein secreted into the maternal circulation reflects the physiological or disease state, and change in the expression level indicates the risk [8]. So far, comparative analysis of proteomics from different sources in different periods of GDM has been conducted in a number of studies [9, 10], showing a great potential of proteomics in GDM research.

In this study, mass spectrometry-based differential proteomics analysis was performed to screen differentially expressed proteins in serum samples between normal pregnancy and pregnancy with GDM. Bioinformatics analysis revealed that most differential regulatory proteins in GDM are related to coagulation function, lipid metabolism, immune response, and inflammation. These proteins can be used as GDM biomarkers and facilitate the early diagnosis and prognosis of the disease. Meanwhile, targeting GDM-related factors could provide new strategies for the clinical treatment of GDM.

## 2. Materials and Methods

### 2.1. Serum Samples

The patients who were admitted to the First Affiliated Hospital of Fujian Medical University from June 2019 to January 2020 were included in the study. According to the medical history and results of the 75 g oral glucose tolerance test (OGTT), that is, the patient can take 75 g of glucose solution orally, compare the blood glucose level with the fasting blood glucose level after two hours. If the fasting blood glucose is greater than 7.0 mmol/L, the blood glucose over 11.1 mmol/L two hours after the oral glucose tolerance test can be considered as diabetes. These patients were divided into the normal pregnant women group (*n* = 8) and GDM pregnant women group (*n* = 12). After written informed consents were obtained, blood samples were collected. 5 mL blood samples was taken and placed in a glass tube without any additives. The blood was clotted for 30 min at room temperature and centrifuged at 3000 g for 10 min at 4°C, and the separated serum was stored at −80°C. The study was approved by the hospital ethical committee.

### 2.2. Protein Extraction

An appropriate amount of SDT lysis buffer (4% sodium dodecyl sulfate, 0.1 M dithiothreitol, and 100 mM Tris-HCl) was added to serum, mixed well, and then bathed in boiling water for 10 min. After centrifugation at 14000 g for 15 min, the supernatant was taken and then filtered using a 0.22 *µ*m centrifuge tube to collect the filtrate. The BCA method was used for protein quantification. The protein samples were divided and stored at −80°C. The protein extraction was performed on serum samples of 12 pregnant women with GDM and 8 normal pregnant women.

### 2.3. SDS-PAGE Electrophoresis

The quality of protein samples was evaluated by sodium dodecyl sulfate polyacrylamide gel electrophoresis (SDS-PAGE). For each sample, 20 *μ*g of protein was dissolved in SDS-PAGE loading buffer (6X) and boiled for 5 min. The protein was loaded on a 12% SDS-PAGE gel, stained with Coomassie Brilliant Blue, and then electrophoresed (constant voltage 250 V, 40 min).

### 2.4. FASP Enzymatic Hydrolysis

200 *µ*g of protein solution was taken from each sample and mixed with dithiothreitol at a final concentration of 100 mM. The mixture was incubated in a boiling waterbath for 5 min and then allowed to cool to room temperature. 100 mM iodoacetamide buffer was added to the mixture, oscillated, and reacted at room temperature in dark for 30 min prior to centrifugation. Subsequently, 4 g trypsin was added to the filtrate, shaken for 1 min, and centrifuged at 37°C for 16–18 h. After being collected, the peptides were desalted using C18 Cartridge, lyophilized, reconstituted with 40 *μ*L of 0.1% formic acid solution, and subjected to quantification.

### 2.5. HPLC Fractionation

The tryptic peptides (Shanghai Yaxin Biological Co., Ltd.) were fractionated by high pH reverse-phase HPLC using the XBridge Peptide BEH C18 column (Waters, 130 Å, 5 *µ*m, 4.6 mm × 100 mm). Briefly, peptides were first separated into 48 fractions with a gradient of 5–45% acetonitrile (pH 10.0) over 40 min and then combined into 12 fractions and dried by vacuum centrifuging.

### 2.6. LC-MS/MS Analysis

The tryptic peptides were dissolved in 0.1% formic acid (solvent A) and then directly loaded onto the Acclaim PepMap RSLC C18 column (Scientific Thermo Fisher, 50 *µ*m × 15 cm). The gradient was comprised of holding at 1% for the first 5 min, an increase from 1% to 28% solvent B (0.1% formic acid in 80% acetonitrile) over 90 min, 28% to 38% for 15 min, and climbing to 100% in 5 min, at a constant flow rate of 300 nL/min on an Easy nLC system (Scientific Thermo Fisher).

The peptides were analyzed by the electrospray ionization tandem mass spectrometry (ESI-MS/MS) in Q Exactive HF-X (Scientific Thermo Fisher) coupled online to the Easy nLC. The electrospray voltage of 2.0 kV was applied. The m/z scan range of primary MS and scanning resolution were set as 350–1500 and 60,000, respectively. Peptides were then selected for MS analysis using NCE setting of 28, and the fragments were detected at a resolution of 15,000. Automatic gain control (AGC) was set at 2e5, while the maximum injection time (IT) and dynamic exclusion duration were set to 45 ms and 30.0 s, respectively.

The original mass spectrometry data were merged and analyzed by Spectronaut Pulsar *X* (version 12, Biognosys AG) to establish a spectral database, Uniprot_HomoSapiens_20386_20180905 (http://www.uniprot.org). For the database search, trypsin digestion was set, with two missed cutting sites allowed. Carbamidomethylation on cysteine (C), was defined as a fixed modification of library search parameters, while variable modifications included oxidation on methionine (*M*) and acetylation on the protein N-terminus. Both precursor and peptide FDR were controlled at 1%. For identification of differentially expressed proteins, the fold changes and *p* value (Student's *t*-test) should be > 1.2 or <0.83 and < 0.05, respectively.

### 2.7. PRM Assays

The parallel reaction monitoring (PRM) method was used to verify the differentially expressed proteins. Peptide separation was performed on the Acclaim PepMap RSLC C18 analytical column using a multistep gradient of B: 2–8% for 1 min, 8–28% for 10 min, 28–40% for 10 min, and 40–90% for 1 min. Then, B was held at 90% for 3 min. A flow rate of 300 nL/min was used, and the analysis duration was 60 min. ESI source settings were the same as above. The PRM analysis included a full MS1 event followed by up to 10 targeted MS2 events. The m/z scan range of MS1 and scanning resolution were set as 350–1500 and 60,000, respectively. AGC target value was set to 3e6, and maximum IT was 45 ms. For MS2, scan settings were 15,000 resolving power, AGC target 2e5, maximum IT 45 ms, normalized collision energy 27 eV, and isolation window was set to 2.0 m/z.

### 2.8. Bioinformatics Analysis

NCBI BLAST+ (ncbi-blast-2.3.0+) was utilized to compare the gene ontology (GO) annotations of differentially expressed proteins with the appropriate protein sequence database, and the top 10 aligned sequences that meet the appropriate *E* value ≤ 1e-3 were retained for subsequent analysis. Functional annotation was carried out using the online Kyoto Encyclopedia of Genes and Genomes (KEGG) database (http://geneontology.org/). Both GO and KEGG pathway enrichment analyses were performed based on Fisher's exact test. In clustering analysis, quantitative data of the target protein set were normalized first. Then, the software Matplotlib was applied to classify samples and protein expression in two dimensions at the same time (Euclidean distance, average linkage clustering). The hierarchical cluster membership was defined by plotting a heat map.

## 3. Results

### 3.1. Protein Identification

Quantitative and SDS-PAGE analyses showed that the protein was of good quality, sufficient, and good in parallelism between samples (Figure S1). Moreover, quantitative normalization was carried out for each group of samples to ensure the accuracy of mass spectrometry results (Figure S2).

A total of 8135 specific peptides and 1152 proteins were identified in all samples. The comparison between the pregnant women with GDM and controls led to an identification of 41 differentially expressed proteins based on the protein identification criteria; among them, 15 were upregulated, while 26 were downregulated in the GDM group (Table 1 and Figure 1).

### 3.2. PRM Verification

To verify the expression levels of differentially expressed proteins, PRM was employed to analyze the expression patterns of 41 target proteins in the same sample. In the experiments, only 12 target proteins were quantified due to restrictions in the characteristics and expression abundance of certain proteins (Table 2). Strikingly, PRM-based verification obtained consistent results with those of the proteomics analysis.

### 3.3. Bioinformatics Analysis

GO annotations were performed to identify biological processes, molecular functions, and cellular components related to the differentially expressed proteins. As shown in Figure 2(a), the main biological processes involve the cellular process, metabolic process, biological regulation, response to stimulus, and immune system process, while the main involved molecular functions and cell components include binding and catalytic activities and extracellular region part, cell part, protein-containing complex, and membrane, respectively. Moreover, GO analysis revealed that the differentially expressed proteins are enriched in either biological processes, such as the metabolism of lipoprotein, fucose, glycoside, and cholesterol, or molecular functions including activities of alpha-L-fucosidase, and arylesterase, and binding of cholesterol and phospholipid or cell compositions such as high-density lipoprotein particle and cytoplasmic vesicle membrane (Figure 2(b)). Meanwhile, the KEGG pathway annotation showed that the differentially expressed proteins are enriched in the cholesterol metabolism, other glycan degradation, and lysosome (Figure 2(c)). As shown in Figure 3, hierarchical cluster analysis of the two experimental groups demonstrated that GDM pathogenesis involves dysfunction of numerous pathways.

## 4. Discussion

Although advanced age, overweight, and obesity have been shown to be risk factors for GDM [11], its pathogenesis remains elusive. To elucidate the molecular mechanism of GDM and to search for potential serum markers for early diagnosis, we identified and quantitatively analyzed the differentially expressed proteins in the serum of pregnant women with gestational diabetes and healthy controls. A total of 41 differentially expressed proteins were identified between the two groups. We further showed that these proteins are correlated with distinct biological processes and signal transduction pathways, suggesting that development of GDM may involve various mechanisms and proteins, including blood coagulation, fibrin clot formation, lipid metabolism, and immune and inflammatory responses.

Under normal physiological conditions, pregnancy leads to activation of the coagulation system and fibrinolysis system, promoting the balance of coagulation function and ensuring the stability of the body's coagulation. Compared with normal pregnant women, pregnant women with GDM exhibit more obvious changes in coagulation and fibrinolysis. The occurrence of diabetes enhances the activation of platelets and coagulation factors [12]. It was reported that the levels of prothrombin time and activated partial thrombin time of GDM patients were significantly lower than those of the nonpregnant group and healthy pregnancy group, whereas fibrinogen and plasminogen levels in GDM patients were markedly increased [13]. Here, we found that alpha-2-macroglobulin (A2MG) and fibrinogen alpha chain (FIBA) were downregulated in the GDM group. A2MG is a broad-spectrum glycosylation inhibitor of various proteases including blood coagulation-related proteases, which is believed to be associated with inflammatory response and coagulant properties [14, 15]. FIBA is chopped up by the protease thrombin to generate monomers that are subsequently polymerized with fibrinogen beta and fibrinogen gamma to form an insoluble fibrin matrix [16]. As one of the main components of blood clots, fibrin plays a major role in hemostasis and thrombosis [17], making pregnant women with GDM more prone to hypercoagulable state. Furthermore, we observed that in the GDM group, coagulation factors *X* and XII were upregulated, whereas coagulation factors including V, XIII, and others were downregulated, albeit no significant difference between the GDM group and controls was present. Collectively, these results suggest that the apparent hypercoagulability of pregnant women is a potential risk factor for GDM patients.

Poor blood glucose control in diabetic pregnant women affects not only the blood coagulation system but also the lipid metabolism [18]. Studies have shown that in patients with poorly controlled GDM, higher concentrations of high-density lipoproteins and higher triglyceride levels were detected in the third trimester and the second and third trimesters, respectively. Another study suggested that APOA-II, APOC3 [19], APOE, and PON1 [9] might be candidate biomarkers for GDM. Consistent with the above studies, we observed significantly higher levels of apolipoproteins APOE and APOC3 in the serum of GDM pregnant women. Moreover, we showed that the level of apolipoprotein APOL1 increased significantly, whereas the levels of cholesteryl ester transfer protein (CETP) and zinc-alpha-2-glycoprotein (ZA2G) decreased markedly. CETP regulates the reverse transport of cholesterol, by which excess cholesterol is removed from surrounding tissues and sent back to the liver for elimination. ZA2G is a novel adipokine related to the lipid metabolism that stimulates lipid degradation in adipocytes and causes extensive fat losses associated with certain advanced cancers [20]. Mracek et al. [21] suggested that ZA2G has a protective effect on the development of obesity and is related to insulin resistance. Together, these results support the role of the lipid metabolism and transport in GDM and suggest its potential for prediction and diagnosis of GDM.

In this study, we identified ectonucleotide pyrophosphatase/phosphodiesterase family member 2 (ENPP2) as the most upregulated protein in the GDM group, which is implicated in obesity-related metabolic phenotypes. It has been reported that increased ENPP2 expression in adipose tissue is closely related to impaired glucose homeostasis and/or insulin resistance [22], while ENPP2 gene regulation affects immune cell population and tissue inflammation in adipose tissue [23]. Although studies have shown that ENPP2 may play a role in induction of parturition [24, 25], the relationship between ENPP2 and the onset of GDM remains to be determined. Given that increased expression of ENPP2 protein may be related to GDM, it needs to be further investigated whether ENPP2 is involved in GDM pathogenesis and can act as a potential biomarker.

In this study, we performed proteomic analysis of maternal serum samples to identify differentially expressed proteins associated with GDM. A total of 41 proteins displayed an expression pattern that was significantly different between pregnant women with GDM and normal pregnant women. Furthermore, bioinformatics analysis suggested that the occurrence and development of GDM may involve multiple biological and pathological processes, such as blood coagulation, fibrin clot formation, lipid metabolism, immunity, and inflammation. Thus, proteins related to the above processes could have potentials as candidate biomarkers for predicting GDM or as intervention targets for preventing the development of GDM.

We need to make a statement, this manuscript had ever been presented as “preprint” in “Research Square,” but which had not been published [26].

## Figures and Tables

**Figure 1:** Volcano plot of differentially abundant proteins (fold change ≥1.2 or fold change ≤0.83 and *p* value <0.05) in the samples between pregnant women with GDM and normal pregnant women.

**Figure 2:** (a) Level 2 statistics of GO function annotations of differentially expressed proteins. (b) GO enrichment analysis of differentially expressed proteins (top 10). (c) KEGG pathway enrichment analysis of differentially expressed proteins (top 10).

**Figure 3:** Hierarchical cluster analysis of differentially expressed proteins between the two different groups, including A (GDM pregnant women) and B (normal pregnant women).

**Table 1:** The differentially expressed proteins identified in the different groups.

Protein names	Accessions	Gene names	Fold change	*P* value
ENPP2	Q13822	ENPP2	2.41009	0.00099
LCAP	Q9UIQ6	LNPEP	2.12435	0.02582
PSG5	Q15238	PSG5	1.85227	0.03598
ADA12	O43184	ADAM12	1.82532	0.02463
UBB; UBC; RS27A; RL40	P0CG47; P0CG48; P62979; P62987	UBB; UBC; RP S27A; UBA52	1.77024	0.01534
HV70D	A0A0C4DH43	IGHV2-70D	1.74216	0.01042
PSG11	Q9UQ72	PSG11	1.60007	0.00165
FIBA	P02671	FGA	1.52207	0.00363
CYTC	P01034	CST3	1.48321	0.01388
APOE	P02649	APOE	1.44068	0.03843
APOC3	P02656	APOC3	1.38564	0.00234
FUCO2	Q9BTY2	FUCA2	1.33303	0.01546
GNPTG	Q9UJJ9	GNPTG	1.32306	0.00226
FUCO	P04066	FUCA1	1.31738	0.03303
APOL1	O14791	APOL1	1.29031	0.00612
PON1	P27169	PON1	0.82963	0.02868
IGLC2	P0DOY2	IGLC2	0.82383	0.03519
IGLC3	P0DOY3	IGLC3	0.82383	0.03519
CR063	Q68DL7	C18orf63	0.81486	0.02107
GELS	P06396	GSN	0.80875	0.00262
ZA2G	P25311	AZGP1	0.80875	0.01114
DDX55	Q8NHQ9	DDX55	0.78727	0.02054
IC1	P05155	SERPING1	0.78424	0.02103
APOA4	P06727	APOA4	0.78039	0.00947
KV315	P01624	IGKV3-15	0.76482	0.02777
LV743	P04211	IGLV7-43	0.73672	0.04679
ECM1	Q16610	ECM1	0.73321	0.01806
A2MG	P01023	A2M	0.71869	0.00313

**Table 2:** PRM quantification results.

Protein names	Accessions	Gene names	Quantification type	PRM	*P* value
ENPP2	Q13822	ENPP2	MS2	2.4777	0.0007
LCAP	Q9UIQ6	LNPEP	MS2	2.1963	0.0232
ADA12	O43184	ADAM12	MS2	1.8293	0.0307
FIBA	P02671	FGA	MS2	1.5337	0.0089
CYTC	P01034	CST3	MS2	1.3124	0.0849
APOE	P02649	APOE	MS1 + MS2	1.4429	0.0438
APOC3	P02656	APOC3	MS2	1.6852	0.0013
APOL1	O14791	APOL1	MS2	1.1492	0.4204
ZA2G	P25311	AZGP1	MS2	0.9674	0.7255
A2MG	P01023	A2M	MS1 + MS2	0.7891	0.0749
SAA4	P35542	SAA4	MS2	0.6903	0.0770
CETP	P11597	CETP	MS2	0.7305	0.1371

## Data Availability

The analyzed data are available for noncommercial use from the corresponding author upon request.

## Supplementary Materials

Supplementary Materials Figure S1. Quality control of protein samples. Quantitative and SDS-PAGE analyses showed that the protein was of good quality, sufficient, and good in parallelism between samples. Figure S2. Before and after quantitative normalization of mass spectrometry data of each group.
